The article "Mitigated Oxidative Stress and Cognitive Impairments in Transient Global Ischemia using Niosomal Selegiline-NBP delivery" was published in 2022. Journal: Behav Neurol.

# Mitigated Oxidative Stress and Cognitive Impairments in Transient Global Ischemia using Niosomal Selegiline-NBP delivery

**DOI:** 10.1155/2022/4825472

**Published:** 2022-04-16

**Authors:** Bahareh Jafari, Mahmoud Gharbavi, Yasamin Baghdadchi, Hamidreza Kheiri Manjili, Javad Mahmoudi, Iraj Jafari-Anarkoli, Shayan Amiri, Mir-Jamal Hosseini

**Affiliations:** ^1^Zanjan Applied Pharmacology Research Center, Zanjan University of Medical Sciences, Zanjan, Iran; ^2^Nanotechnology Research Center, Ahvaz Jundishapur University of Medical Sciences, Ahvaz, Iran; ^3^Zanjan Pharmaceutical Biotechnology Research Center, Zanjan University of Medical Sciences, Zanjan, Iran; ^4^Neurosciences Research Center, Tabriz University of Medical Sciences, Tabriz, Iran; ^5^Department of Anatomical Sciences, School of Medicine, Zanjan University of Medical Sciences, Zanjan, Iran

## Abstract

Stroke is the most common reason for adult disabilities and the second ground for death worldwide. Our previous study revealed that selegiline serves as an alternative candidate in transient hypoxia-ischemia. However, aggressive and restless behavior was observed in stroke-induced rats receiving 4 mg/kg selegiline. In comparison, 1 mg/kg selegiline could induce negligible therapeutic effects on mitochondrial dysfunction and histopathological changes. Therefore, we designed oral noisome-based selegiline attached to 4-(4-nitrobenzyl) pyridine to improve transient global ischemia by attenuating cognitive impairments, oxidative stress, and histopathological injury. The investigation was performed in transient hypoxia-ischemia-induced rats by oral administration of nanoformulation containing selegiline (0.25-1 mg/kg) for 4 weeks (3 times a week). Novel object recognition (NOR) was considered to evaluate their cognitive dysfunction. Oxidative stress parameters and brain histopathological assessments were determined following the scarification of rats. Outstandingly, our data demonstrated slower selegiline release from niosomes relative to free drug, which was also in a controlled manner. Our data confirmed significant improvement in cognitive behavior in the NOR test, an increase in glutathione level and total antioxidant power, a decline in MDA and protein carbonyl level, as well as a decreased number of dead cells in histopathological assessment after being exposed to (0.5-1 mg/kg) selegiline-NBP nanoformulation. These data manifested that the selegiline-NBP nanoformulation (0.5-1 mg/kg) could significantly reduce oxidative damage, cognitive dysfunction, and histopathological damage compared to transient hypoxia-ischemia rats, which is 20 times lower than the therapeutic dose in humans. Therefore, the proposed nanoformulation would be capable as an alternative candidate without side effects in stroke.

## 1. Introduction

Stroke is a devastating neurological condition, which deteriorates the quality of life and causes mortality and disability throughout the world [1]. Unfortunately, the resulting burden of stroke on society is growing with the increase in its incidence [2, 3]. Few patients are eligible for the immediate restoration of cerebral blood flow by thrombolytic agents since it is effective only in a limited time window after stroke onset and only helps open occluded cerebral vessels [4]. In the ischemic stroke condition, pathological damage is observed following inflammation, oxidative stress, cell death signaling induction, and edema which is correlated to blood-brain barrier (BBB) disruption [5]. Therefore, it is highly required to represent a neuroprotective agent with the capability of preventing neuronal damage and sharpening restoration [6].

Although different therapeutic agents have been proposed or are being examined, the ideal drug was not recognized as an effective neuroprotective therapy in stroke patients [7]. Selegiline has shown promising effects for recovery after stroke, particularly in cognitive functioning. Significant improvement was evident in cognitive performance after two and six weeks of selegiline intake (10 mg/day). The domains of attention and executive functions are also recognized as the most beneficial parts [1]. Good evidence supports the clinical neuroprotective/neurorescue capacity of selegiline with regard to the pathogenic role of “oxidative stress.” However, the clinical application of MAOIs may be restricted by the possible adverse effects of restlessness and insomnia [8, 9].

The previous studies proposed that selegiline, which can be an alternative drug in the treatment of transient global ischemia, acts through MOA-B inhibition, antioxidant effect, and production of L-methamphetamine (METH) in the metabolic pathway of selegiline [10]. Rau et al. revealed that a low dose of L-METH 12 hours after stroke mediates neuroprotection via positive effects on cognition behavior [11, 12]. The neuroprotective effects of L-METH against stroke injuries have been demonstrated through the activation of PI3K, phosphorylation of protein kinase 3, increasing phosphorylation of AKT, and upregulation of antiapoptotic BCL-2 gene [13]. Our previous study showed that a shortage of physical and mental dependence is the advantage of selegiline to L-METH in stroke therapy [10].

Unfortunately, we observed some behavioral abnormalities such as aggressiveness and restlessness during the treatment periods with higher doses of selegiline, which can be considered a limitation of our previous work. Thus, we decided to solve this dosage limitation problem by designing a nanoformulation composed of 4-(4-nitrobenzyl) pyridine or (NBP) as a specific 3A4 metabolic inhibitor coupled to selegiline. Furthermore, the development of drug delivery to the brain attracts a great deal of attention for therapeutic purposes of stroke via enhancement of the bioavailability and providing a controlled therapeutic activity for a prolonged period [14]. Niosomes the nonionic surfactant vesicular systems are of great interest for the formulation of drugs since encapsulation in niosomes can enhance stability and bioavailability with the facile synthesis method in the laboratory [15]. In this work, we decided to examine the protective effects of oral nanoformulated selegiline coupled with NBP against transient global ischemia in rats.

## 2. Material and Methods

### 2.1. Materials

All the materials used in this investigation were purchased from Sigma-Aldrich (Germany).

### 2.2. Niosome-BSA Preparation

The thin-film hydration process (handshaking technique) was applied in order to fabricate niosomes, as formerly reported [16]. In summary, in a round-bottomed flask, 300 mg of surfactant mixture (Tween 80 and Span 80) and 80 mg cholesterol, as well as 8.56 *μ*g NBP were dissolved in chloroform. Next, the organic solvent was detached at 60°C under reduced pressure by a rotary evaporator at 150 rcf to form the thin lipid layer. Then, BSA (100 mg) and selegiline (50, 25, or 12.5 mg) were dissolved in 5 mL double distilled water under continuous stirring (600 rpm) at room temperature for 15 min. Subsequently, 5 mL of the obtained solution was added to the flask and mixed by vortex for 1 min. The mixture was then emulsified by 30 min of sonication in a water bath at 50°C [17].

## 3. Physicochemical Characterizations

### 3.1. Morphology Analysis

Scanning electron microscopy (SEM) was performed to study the niosome nanoformulated morphology. For this reason, gold was applied to coat lyophilized niosomes. Then, at a stepping up 15 kV voltage, niosomes were witnessed using SEM (MIRA TESCAN, Czech Republic).

### 3.2. Evaluation of Niosome Size and Zeta-potential

A nano-/zeta-sizer (Malvern Instruments, Worcestershire, UK, model Nano ZS) was used to determine the mean particle size, size distribution, and surface charge of niosomes by dynamic light scattering (DLS). For this reason, ultrapure water (1.5 mL) was added to 0.5 mL of samples containing niosomes to make it diluted.

### 3.3. FT-IR Analysis

In order to obtain spectra of selegiline, BSA, and niosome-BSA, the FI-IR analysis was carried out using pellets of KBr and the infrared microscope (Spectrum Two, USA). Approximately, 1.25 mg prepared samples was mixed with 250 mg KBr and passed in plate form. The scanned range for FTIR spectra was between 400 and 4000 cm^−1^.

### 3.4. Electrical Conductivity Capacity

Electrical conductivity (EC) for the as-prepared niosomes was determined with the electrical conductivity meter Metrohm Model 712 at room temperature and in triplicate.

### 3.5. Index of Refraction

Niosome samples were tested in terms of their ability to reflect light. For this reason, refractometer M46.17/63707 (Higler and Walts Ltd., England, UK) was applied, and a droplet from the solution was poured onto the slide at 25°C [18].

### 3.6. Estimation of Limpidity

Percent transmittance of the as-prepared samples was evaluated at 633 nm with a spectrophotometer (Shimadzu, UV-160, Japan). The experiment was performed with three repeats for each sample and double distilled water as a blank sample [19].

### 3.7. Measurement of pH

First, the pH meter was calibrated using buffer solutions with pH 4.0, 7.0, and 9.0. After that, the pH values of nanoformulated samples were determined using Corning 220 pH meter (Cole-Palmer, Teddington, UK) at room temperature. Indeed, the goal of this test was to explore the impact induced by niosomes and confirm whether selegiline existed at different pH or not. Furthermore, it aimed at providing a platform to compare the obtained data with that of blood plasma. The pH value of niosomes was read three times for each sample, and the averages were calculated [20].

### 3.8. Rheological Behavior

A viscometer (Brookfield Viscometer LTD) was applied to study the rheological features of niosomes and niosomes encapsulated with selegiline [21]. To this end, 1.5 mL of niosomes samples was put in the reading plate, and the superfluous sample was discarded. Next, the Brookfield Viscometer LTD Software was used to obtain data.

### 3.9. Entrapment Efficiency

Selegiline entrapment efficiency (EE %) in prepared niosomes was determined from the nonentrapment-free drug as described method [22]. Briefly, after preparing niosomal dispersion, the unentrapped drug was separated by centrifugation using pH 7.4 phosphate buffer for 15 min at 17,000 rpm. Experiments were carried out at least three times to verify the separation of all nonentrapment-free drug niosome formulations. The resulting solution was analyzed by UV spectrophotometer (Thermo Fisher Scientific, *USA*, Madison, model GENESYS™ 10S) at wavelengths of 205 nm for the total amount of entrapped drug. The selegiline entrapment efficiency (EE %) was assessed in accordance with the formula presented hereunder:

(1) $$\begin{array}{c} Entrapment\text{ Efficiency }\left(\text{EE}\%\right)=\frac{Amount\;\text{of }Drug-\text{Non }entrapment\;\text{of }Drug}{Amount\;\text{of }Drug}\times 100. \end{array}$$

### 3.10. *In Vitro* Stability of Niosome Samples in SGF and SIF

Physical stability of fabricated niosomes was verified by examining Z-average (nm), polydispersity index (PDI), and Z-potential (mV) in SGF and SIF media, after 40 min and 6-hour incubation time, respectively. During the experiment, samples were kept in bain-marie and gently shaken at 37°C. Three repeats were done for each sample. Simulated gastric fluid (SGF) and simulated intestinal fluid (SIF) were primed as stated by USP specifications. Niosome samples (free-niosomes and niosome-selegiline) were incubated in SGF (0.2 g NaCl, 0.7 mL HCl, and triple distilled water up to 100 mL, pH 1.2) or SIF (0.680 g KH_2_PO_2_, 0.616 g NaOH, and triple distilled water up to 100 mL, pH 6.8).

### 3.11. In Vitro Studies of Drug Release in Different Media

The *in vitro* release of selegiline from niosomes was performed in three media: phosphate-buffered saline (PBS), SIF, and SGF. The experiments were done under immersed settings at 37°C for 144 hours in PBS with pH 7.4, 6 hours in pH 6.8 solution (SIF) and, 2 hours in pH 1.2-buffer solution (SGF). Dialysis tubing (molecular weight cut off − >12, 000, Hi media) earlier drenched overnight in the receptor medium was on Franz's Diffusion cell assembly. 1 mL from niosome-selegiline was suspended in 1 mL of the preincubated reaction mixture of PBS, SIF and, SGF, put in dialysis bags (molecular weight cut off − >12, 000), and they were incubated in 20 mL of an incubated mixture of PBS with pH 7.4), SIF (pH 6.8) and SGF (pH 1.2), and were smoothly shaken at 37°C with three repeats. Then, at arranged time intervals, 0.5 mL of the release solution was discarded and replaced by equal fresh media. The release behavior of selegiline from niosomes was determined using UV spectrophotometry at 205 nm consistent with the standard calibration curve [23].

The *in vitro* selegiline release data (at pH 7.4) were evaluated by fitting them to different kinetic models, for estimating kinetics and mechanisms of selegiline release (Table 1). The ideal kinetic model was accepted according to the least values for the mean squared error (MSE) and Akaike's information criterion (AIC).

### 3.12. Hemocompatibility

Hemolysis assay is vital to guarantee the compatibility of the proposed system with the components of blood. Hemolysis is defined as when the erythrocyte membrane has been damaged. Hence, the level of hemolysis induced by niosomes samples was determined using the previously stated hemolysis assay approach [24]. Human blood for the biocompatibility assay was taken with ethical consent and kept in heparin-containing pipes. Then, the fresh blood was centrifuged at 4000 rpm for 5 min. Next, the supernatant was detached, and red blood cells (RBCs) were obtained after three items of washing with sterile PBS. After that, RBCs were resuspended in isotonic PBS to become diluted to 10% of their primary concentrations, i.e., various concentrations of ME samples (50-300 *μ*g/mL). Afterward, 1% sodium dodecyl sulfate (SDS) as positive control and 500 *μ*L PBS as negative control were used. 200 *μ*L RBC was then added to each sample and was incubated in a bain-marie at 37°C. After 4 hours, samples were centrifuged at 4,000*g* for 10 min. Lastly, the absorbance of the supernatant was read at 541 nm by a plate reader [25]. The test was performed in three repeats. The subsequent equation was applied to calculate the percentage of hemolysis:

(2) $$\begin{array}{c} Hemolysis\;\left(\%\right)=\frac{\;A_{treated\;sample}-A_{negetive\;control}\;}{\;A_{positive\;control}-A_{negetive\;control}}\times 100. \end{array}$$

*A*_treated sample_ characterizes the mean absorbance of niosomes (test). Likewise, *A*_negative control_ and *A*_positive control_ symbolize the mean absorbance of negative and positive control, in turn.

### 3.13. Animals

Male Wistar albino rats weighing 220–250 g were housed in line with the standard laboratory conditions and were treated under the protocol approved in agreement with NIH guidelines (NIH Publications No. 8023, revised 1978).

### 3.14. Transient Global Ischemia Induction

The rats were severely anesthetized with IP injection of ketamine and xylazine (100 and 8 mg/kg, respectively). Next, the anesthetized animals were sited supine, and after shaving their neck, the skin was cleansed with betadine and wetted with 70% ethanol. In the surgery, both common (right and left) carotid arteries were wide-open and separated from the vagus nerve by midline incision on animals' necks. After that, both of them were shortly closed by vascular microclips. The clamps were then removed 20 min postclamping, so with reperfusion, the incision spot was saturated [10].

### 3.15. Study Design

Rats were randomized into 7 groups (*n* = 12 animals per group) and were treated as following procedures: 1 control that only received normal saline (as a carrier of selegiline); Group 2: nonischemic rats received only noisome+NBP as a specific inhibitor of CYP 450/2B6; Group 3: nonischemic rats received 1 mg/kg of selegiline three times each week for four weeks; Group 4: stroke-induced rats; and Groups 5, 6, 7: ischemic rats received selegiline (0.25, 0.5, and 1 mg/kg) in niosomal selegiline-NBP structure three times each week for four weeks. Towards the end of the treatment duration, the behavioral assessment was performed on rats between 10 : 00 AM and 2 : 00 PM. The effective dose of L-deprenyl (selegiline) for inducing therapeutic impacts on humans is 10 mg/day (5 mg PO at breakfast and 5 mg at lunch) which is equal to 1.6 mg/kg/day in rats due to higher metabolism and calculation from surface area ratio. Besides, we treated rats only three times in the week after, and practically, the protective effects of 0.25 to 1 mg/kg from L-deprenyl were tested in animals. Finally, animals were decapitated and their brain was dissected on an ice-cold plate, frozen abruptly in liquid nitrogen, and maintained in a -80°C freezer for biochemical experiments (Figure 1). The dissected hippocampus in each group was immersed in 10% formalin for histopathological assays.

### 3.16. Novel Object Recognition (NOR) Test

The rodents' aptitude to identify a novel object is measured by the natural propensity of the animal to devote more time to discovering the unfamiliar object than the usual one, which has been helpful to study memory functions in rodents as described by previously published method [10]. The rodents are normally inclined to devote more time to discovering the unfamiliar thing in the initial moments of the test phase. The apparatus, which is used in the NOR task, includes an open box made of Plexiglas (70 × 70 × 30 cm). In this experiment, rats were passed through three steps. Firstly, they spent 15 min of acclimatization in the vacant apparatus two days before starting the test. After 24 h, two equal objects were set in the apparatus at equal distances from the rat and the animal was freed to discover them for 10 min. After that, the rats were returned to cages. In the third step, rats were transferred again into the apparatus after 24 h. In this step, they were provided with one acquainted object and one new object with diverse shapes and colors at the same distances to discover them for 3 min. The data obtained by this test can be used for calculating the discrimination index (DI). It gives rise to discrimination between the novel and familiar objects and applies the variance in exploration time for a familiar object, but then dividing this value by the total amount of exploration of the novel and familiar objects (DI = (*T* novel − *T* familiar)/(*T* novel + *T* familiar)).

### 3.17. Glutathione (GSH) Assay

The amount of reduced glutathione was determined using Ellman's reagent (DTNB) reduction by spectrophotometric assay at the wavelength of 412 nm, which presented *μ*mol/gr tissue [26, 27]. Briefly, 100 mg of tissue was mixed with 1 mL of EDTA (0.02 M) and 1.5 mL TCA (10%W/V) in a homogenizer. After that, 1.25 mL of phosphate buffer (0.4 mol/L) and 0.25 mL of DTNB indicator (0.8 mg/mL; pH = 8.9) were added to 0.5 mL of supernatant, vortexed superbly to measure the absorbance of developed yellow color at 412 nm.

### 3.18. MDA Assay

Briefly, 0.25 mL sulfuric acid (0.05 M) was added to 0.2 mL of homogenate sample (100 mg), and 0.3 mL of TBA 0.2% was then added to tubes and put in a bain-marie for 30 min. Afterward, the tubes were moved into ice and 0.4 mL of *n-*butanol was added to each tube and then centrifuged at 3500×*g* for 10 min [28]. The MDA level made in each sample was obtained by reading the absorbance of the supernatant at 532 nm on an ELISA reader. The test was done using tetramethoxy propane (TMP) as the standard to gain MDA content in *μ*mol/g tissue.

### 3.19. Protein Carbonyl Assay

This test is reliable for revealing protein oxidation using the spectrophotometric method at 365 nm with DNPH (2,4-dinitrophenylhydrazine) reagent according to the conventional technique [29]. In brief, 100 mg of tissue was homogenated in 0.5 mL of 20% (*w*/*v*) TCA and set at 4°C for 15 min. Later on, 0.5 mL of 0.2% DNPH was added to precipitates, as well as 0.5 mL of NaOH (2 M) as control. After 1 h incubation at room temperature, followed by vortex in 5 min intervals, 0.5 mL of TCA (20%) was added to precipitate proteins. All samples were centrifuged, and after three washes with 1 mL ethanol-ethyl acetate, they were dissolved in 0.2 mL of guanidine hydrochloride (6 M). Finally, carbonyl content expressed as nmol/g tissue was obtained by reading the absorbance of the samples at 365 nm wavelength.

### 3.20. Ferric-Reducing Antioxidant Power (FRAP) Assay

The total antioxidant potential stated as mmol/g tissue was estimated by a sensitive reagent of TPTZ. For this reason, the absorbance at 593 nm was measured. The escalation in absorbance value was indicative of the antioxidant activity by the generated ferrous ions following the previous investigation [30].

### 3.21. Histopathological Assays

The hippocampal samples obtained from rats studied for 72 hours were fixed in 10% formalin, followed by processing of sample tissue for the hippocampus. Next, they were sectioned at 5 *μ*M and stained with hematoxylin and eosin (H&E) and studied under a light microscope (Olympus BX51). At last, photos were captured by a camera attached to the microscope with 400x magnitude. 5 slices were randomly selected per rat, and neurons of the hippocampus were counted to find out how many normal and dead neurons existed in the CA1 area of the hippocampus.

### 3.22. Statistical Analysis

SPSS software, version 16, was applied for the data analysis of this work. One-way ANOVA test followed by the Tukey test (*P* < 0.05) was used to verify statistical significance. Further, G power software (ver.3.1.7, Franz Faul, Universitat Kiel, Germany) was used for the estimation of sample size. Results were stated as mean ± standard deviation (SD), while p < 0.05 represents statistical significance.

## 4. Results

### 4.1. Preparation of Niosome-BSA

In the current work, the thin-film hydration method was modified to some extent, where niosomes were coated using BSA. The BSA containing a negatively charged protein at pH 7.4 was used as a stability agent for niosomes. It was seen that the coating of BSA on the surface of niosomes provides excellent properties and biocompatibility for these nanostructures and allows their use as a hydrophilic drug carrier [31].

### 4.2. Morphological Characterization of Niosomes

SEM image of BSA coated niosome formulation is shown in Figure 2. Our results indicated that the suggested niosome formulation had homogeneous spherical morphology, and the surface of niosomes is smooth as expected.

### 4.3. FT-IR Analysis

FT-IR spectra were step by step recorded to approve the presence of components in the formulation. As seen in Figure 3, FT-IR spectroscopy was used to determine the compositions of niosomes, selegiline, and niosome-selegiline. The characteristic absorption peaks of niosomes at 1700 and 3400 cm^−1^ were indicative of a carboxylic acid functional group (C=O) and hydroxy group, respectively [32]. Also, in the FT-IR spectrum of pure selegiline, HCl was characterized by absorption peaks at 2942, 1464, 1093, and 698 cm^−1^, which show the attendance of C-H stretching vibrations at the end of the aliphatic chain, C-N bending, and -N-bending fluctuation, respectively [33]. Accordingly, the presence of characteristic peaks of all the existed components of niosomes (Figure 3(a)) and selegiline (Figure 3(c)) in the FT-IR spectra of niosome-selegiline (Figure 3(b)) confirms the successful encapsulation of selegiline to niosomes.

### 4.4. Determination of Particle size and Zeta-potential

Niosomes and niosome-selegiline size and zeta-potential are shown in Figure 4. It has been reported that particles smaller than 200 nm could improve the stability, bioavailability, and biological properties of drugs, such as their pharmacokinetics and biodistribution [34]. In the current study, the average size of niosome samples was around 118.8 to 142.9 nm, confirming the capability of nanoparticles for oral drug delivery. On the other hand, the amount of bioavailability may rely on the size of the particles. As typical, bioavailability improved with a decrease in particle size [35]. In addition, the zeta-potential of samples are ranged from -10.5 to -13.8 mV. Negative zeta-potential is attributed to hydroxyl groups of surfactants and the cosurfactant, which contain oxygen atoms with high electronegativity [36].

### 4.5. Physicochemical Characterizations

As it is obvious in Table 2, the physicochemical factors of niosomes samples, such as ECM, RI, pH, and %transmittance, were determined. The EC coefficient, RI, and %transmittance were extremely sensitive to both factors of temperature and composition. The EC coefficient, RI, and %transmittance of niosomes samples were recorded at 1.32-1.98 m.s/cm, 1.11-1.22, and 37-42%, respectively. The EC coefficient of niosomes was greater than that of niosome-selegiline, which is associated with the presence of selegiline that may decrease the percentage of water in the sample [37]. The refractive index (RI) of the niosome-selegiline was higher than niosome sample. In light of the arguments discussed before, the RI of the niosome samples is as same as water's RI (1.33).

Likewise, the decreased transmittance of samples was attributed to the surfactant and cholesterol present in the formulation. The pH value of niosomes and niosome-selegiline was between 5.41 and 6.23. The pH value of the niosome-selegiline was higher than that of niosomes, which might be owing to the existence of selegiline inside niosome structure. The integrity of particle structure and the probability of aggregation were estimated to delineate the physical stability of samples. Hence, size monitoring of the samples was performed for three months. It is obvious in Figure 4(a) that the Z-average of T-ME and T-BSA-ME has not risen dramatically in the measurement duration. The efficacy of selegiline encapsulation in niosomes was calculated by applying standard calibration curve in the dose range of 30-120 *μ*g/mL. Furthermore, the correlation coefficient, the limit of detection (LOD), and the limit of quantification (LOQ) were 0.9967, 1.13 *μ*g/mL, and 3.79 *μ*g/mL, correspondingly. Besides, UV-VIS spectrophotometry at 205 nm revealed that selegiline encapsulation in niosomes has an efficacy of over 67.32%.

### 4.6. Rheological Performance

The significance of rheological analysis lies in investigating structural properties, system stability, handling, storage, and pipeline transportation of niosome samples [38, 39]. The shear stress and viscosity as a function of the shear rate for the niosomes and niosome-selegiline are depicted in Figure 5(b). As indicated, at lower shear rates (˂50 S^−1^), the shear stress increased instantly. Shear stress for samples was decreased gradually by increasing the shear rate, which was approximately constant at high shear rates (>100 S^−1^). Accordingly, non-Newtonian viscous behavior is apparent in all samples.

### 4.7. Gastrointestinal Stability of Niosome Formulations

Simulated gastric fluid (SGF) and simulated intestinal fluid (SIF) was primed in accordance with the United States Pharmacopoeia [40]. The SGF and SIF medium was prepared with pH 1.2 and pH 6.8, respectively. The stability of niosome samples in SGF/SIF was evaluated by DLS measurements. Hence, particle size, PDI, and zeta-potential values were examined before and postincubation with SGF and SIF media. According to the results shown in Table 3, it can be concluded that niosomes are stable in SGF and SIF.

### 4.8. Blood Compatibility Assay

For biomedical applications, niosomal system is in close contact with body tissues and cells, so it is essential to guarantee their biosafety in advance. To this end, the minimal hemolytic effect of niosome samples on human RBCs should be assured.  Figure 6(a) shows the biocompatibility of samples was evaluated at a 50-300 *μ*g/mL dose range. The supernatant absorbance at 540 nm (hemoglobin) was measured using Eppendorf Bio Photometer to ascertain the hemolytic activity of the samples [24]. The hemolytic activity of niosomes and niosome-selegiline in different mass concentrations was between 7.27-12.69% and 5-10.4%, correspondingly. The hemolytic activity of niosomal systems can be attributed to the present surfactant. An increased level of surfactant leads to increased hemolysis [41].

### 4.9. Drug Release and Kinetic Study

The dialysis approach is a widespread and flexible technique to evaluate the release behavior of a drug in nanoformulation [42]. The profile of selegiline release from niosomes was studied using this method. Selegiline release from niosomes at buffer solutions (pH 7.4), SGI media (pH 1.2), and SIF media (pH 6.8) is shown in Figures 6(b)–6(d). The cumulative selegiline release from niosomes and free-selegiline drug after 24 hours at pH 7.4 was 27.1% and 85.46%, respectively.

For SGI and SIF, the cumulative selegiline release from niosomes after 2 and 5 hours was 40.17 and 34.87%, respectively. As expected, the drug release from niosome nanocarrier gave slower drug release compared with the free drug in buffer saline, SGF, and SIF media. In addition, niosome formulation released selegiline in a controlled-release mode.

The results gained from empirical data of selegiline release (at pH 7.4) were well suited to different mathematical kinetic models, as indicated in Table 4. The *R*^2^, AIC, and MSE values of the Weibull model showed good fitness with experimental data in niosome-selegiline and free-selegiline at pH 7.4 media.

### 4.10. The Impact of Selegiline-NBP Nanoformulation on Behavioral Distress in the NOR Test

The data obtained from the NOR test exhibited a significant decrease in discrimination index in the global ischemia-induced rats relative to control (nonstroke condition) as these rats were less interested in exploring and learning about the novel object. One-way ANOVA demonstrated significant alteration between different treated groups in cognitive and learning memory in the behavioral test (*F* (7, 53) = 47.859; *P* < 0.001; Figure 7). Post hoc analysis revealed a significant difference in discrimination ratio between nonstroke animals (control) and stroke-induced rats (*P* < 0.001). However, the animals treated with niosomes containing NBP and niosomes containing selegiline+NBP did not show any significant difference in discrimination ratio after 28 days of oral administration compared to the control rats (*P* > 0.05). On the other hand, stroke-induced rats which were then treated with niosomes containing selegiline+NBP (.25, 0.5, and 1 mg/kg) showed that discrimination scores have significantly increased compared to stroke-induced rats and reached the control level (*P* < 0.001; Figure 7).

### 4.11. The impact of Selegiline-NBP Nanoformulation on Glutathione (GSH) Level

Alteration in GSH level as the well-known antioxidant biomarker was assessed. The present data obtained from the brain of rats revealed that animals treated with niosomes containing NBP+selegiline significantly increased the GSH level compared to stroke-induced rats (*F* (7, 53) = 56.766; *P* < 0.001; Figure 8). Indeed, there was a significant decrease in glutathione (GSH) amount in stroke-induced rats compared to normal or nonstroke animals (*P* < 0.001; Figure 8). Then, niosomes containing NBP+selegiline (0.5 and 1 mg/kg) in stroke-induced rats significantly raise the GSH level compared to stroke rats (*P* < 0.001). On the other hand, niosomes containing NBP+0.25 mg/kg of selegiline in stroke-induced animals were not able to reverse GSH to the normal level or similar to nonstroke rats (*P* > 0.05; Figure 8). Also, no significant difference was observed in the GSH level of the rats treated with niosomes containing NBP alone and selegiline (1 mg/kg) compared to the control or nonstroke rats)*P* > 0.05).

### 4.12. The Impact of Selegiline-NBP Nanoformulation on MDA Level in the Brain

MDA as a biomarker for lipid peroxidation was measured by the TBARs method in brain tissues of all groups. Our data revealed that treatment of animals with niosomes containing NBP+selegiline significantly decreased MDA levels compared to stroke-induced rats (*F* (6, 14) = 72.404; *P* < 0.001; Figure 9). We observed substantial change in MDA levels between selegiline-treated groups, normal (nonstroke), and stroke-induced rats (*P* < 0.001; Figure 9). Moreover, animals that received niosomes containing NBP alone or selegiline (1 mg/kg) do not show a significant difference in MDA level compared with control rats (*P* > 0.05). Whereas the stroke-induced rats that were treated with niosomes containing NBP+selegiline (0.25, 0.5, and 1 mg/kg) showed a significant decrease in MDA level compared to stroke-induced rats (*P* < 0.001). It can be inferred from these results that niosomes containing selegiline (0.25 mg/kg)+NBP could significantly reduce the MDA level in stroke-induced rats, but it could not reverse it to the normal level in control or nonstroke rats.

### 4.13. The Impact of Selegiline-NBP Nanoformulation on Protein Carbonyl Level

As shown in Figure 10, protein carbonyl as an indicator of protein oxidation illustrated that treatment of animals with niosomes containing NBP+selegiline significantly decreased protein carbonyl levels compared to stroke-induced rats (*F* (6, 14) = 150.837; *P* < 0.001). Protein carbonyl was significantly increased in stroke-induced rats relative to that of control or nonstroke animals (*P* < 0.001; Figure 10). There was a significant difference between the treatment of stroke-induced animals with niosomes containing NBP+selegiline (0.5 and 1 mg/kg) in comparison with stroke-induced rats (*P* < 0.001). However, niosomes containing NBP+selegiline (0.25 mg/kg) in stroke-induced rats did not indicate any significant difference in protein carbonyl amount compared to stroke-induced rats. Besides, treatment of normal rats with niosomes containing NBP or selegiline did not show any significant change in protein carbonyl compared to the control or nonstroke rats (*P* > 0.05; Figure 10).

### 4.14. The impact of Selegiline-NBP Nanoformulation on FRAP Level

Figure 11 clearly shows a significant rise in FRAP level as an antioxidant power in the brain of animals treated with niosomes containing NBP+selegiline compared to stroke-induced rats (*F* (6, 14) = 41.437; *P* < 0.001). Statistical analysis showed a significant decrease in FRAP level in stroke-induced rats compared with that of the control group. We observed that there was no significant difference in FRAP amount between animals treated with niosomes containing NBP or selegiline (1 mg/kg) compared to control rats. Afterward, the effects of niosomes containing NBP+selegiline (0.25, 0.5, and 1 mg/kg) were assessed in stroke. As shown in Figure 11, FRAP levels in stroke-induced rats which received niosomes containing NBP+selegiline (0.5 and 1 mg/kg) were increased to 422 ± 22 and 549 ± 13.6 mM compared to stroke-induced rats (250.8 ± 24.5 mM). But, niosomes containing NBP+selegiline (0.25 mg/kg) in stroke-induced rats did not yield a significant increase in FRAP levels compared to stroke-induced animals for improving ischemia-reperfusion damage in the brain.

### 4.15. Histopathological Assessment

As indicated in Figure 12, our histological studies in the CA1 area of the hippocampus manifest an increased number of neuronal death in stroke-induced rats compared to control rats. However, the number of dead cells decreased following niosome-selegiline (0.25, 0.5, and 1 mg/kg) treatment in ischemic animals relative to nontreated ischemic ones. Besides, a decrease in the number of dead cells following 1 mg/kg of selegiline in stroke-induced rats was obvious compared to stroke animal rats in this study.

## 5. Discussion

Cerebral ischemia causes neuronal damage in the hippocampus, which leads to disturbance in cognitive behavior. Numerous studies and our previous research have shown the involvement of oxidative stress in cerebral ischemia such as an increase in ROS level and decline in intracellular enzymatic and nonenzymatic antioxidant defense systems [43, 44].

Interest in selegiline as a possible neuroprotective agent has been expanding in the past few years, primarily because of exciting findings by a wide variety of *in vitro* and *in vivo* investigations [45]. Our previous data showed that selegiline is able to effectively decrease neuronal death in the hippocampus (HIPP), under ischemic conditions [10]. It is postulated that the neuroprotective properties of selegiline are associated with MAO-B inhibitory activity, propargylamine group, and the capability of L-methamphetamine (the metabolite) to attenuate brain injury. Other previous studies confirm that [26, 46] low doses of METH in animal models can reverse the cognitive impairment in the recognition of novel objects from familiar ones [47].

Moreover, our previous investigation revealed that although 4 mg/kg selegiline could entirely reverse mitochondrial dysfunction and cognitive behavior, it caused aggressiveness and impaired social interaction [10]. Hence, to address the challenges regarding optimized therapeutic effects of selegiline, here, we have proposed the application of selegiline-NBP nanoformulation to attenuate oxidative stress and cognitive impairments in the treatment of transient global ischemia. Due to the hydrophilic nature and adverse effects of selegiline in high doses (≥ 4 mg/kg), we designed the surfactant-based nanocarrier for the treatment of transient global ischemia. Also, it has been demonstrated that selegiline is metabolized to (−)-methamphetamine and des-methyl deprenyl [48]. Several studies have indicated that the effects of selegiline on the brain involve biotransformation of the drug into these two metabolites that both can induce neuroprotective effects. Nevertheless, metabolite levels are quite low compared to the initial selegiline dose. Therefore, for beneficial effects, higher doses of selegiline are required [49–51]. Hence, to decrease selegiline dosage and solve the aforementioned problem, NBP was placed on the hydrophobic surface of niosomes as it brings specific inhibition of CYP 450/2B6 for the higher transformation of selegiline to L-METH [52]. In this way, the metabolism line to produce des-methyl-selegiline will be blocked, resulting in higher production of the other metabolite, which is more important in terms of neuroprotective effects. Thus, it is supposed that lower doses of selegiline (≤1 mg/kg) can induce higher neuroprotective effects.

We aimed to evaluate the effectiveness of the proposed nanoformulation following cognitive-behavioral tests, as well as biochemical assay and histopathological investigation. In the present study, the thin film hydration technique was applied for niosome preparation through a simple method. It was made by dissolving surfactant mixture (Tween 80 with high HLB value, Span 80 with low HLB value) with cholesterol in an organic solvent in a flask, which results in allowing them to run together, and subsequently make a stable formulation [53]. Tween 80 and Span 80 were chosen as a surfactant mixture owing to low toxicity and biocompatibility [54, 55]. The mean average size of our synthesized NPs was lower than 200 nm, with a polydispersity index (PDI) in the range of below 0.4, indicating good size and uniformity in the distribution of nanoparticles size. The stability of nanoparticles was confirmed by zeta-potential (±30 mv). Furthermore, the successful encapsulation of selegiline in noisome structure was verified by FT-IR with a loading rate of 67.32% for selegiline. Our results indicated that the stability of niosome formulations did not showed significant changes in the size, PDI, and zeta-potential after 140 hours in the physiological pH (7.4), 1 hour in stomach pH (1.2), and 5 hours in intestinal pH (6.8). It can be concluded that the suggested niosome formulation is an excellent nanocarrier for selegiline delivery with a controlled release manner and a good therapeutic outcome.

The therapeutic effects of selegiline, when delivered by this carrier, were assessed by measuring the cognitive behavior and oxidative stress parameters in the rat's brain. The data obtained by the NOR test [56] demonstrates that selegiline nanoformulation is effective in the process of recognition, memory, and learning. Our data pointed out that rats treated with niosome-NBP-selegiline (0.25-1 mg/kg) revealed a higher discrimination index compared to the transient global ischemia and similar to normal rats. These data suggested that niosome formulation could more effectively enhance learning and recognition memory in transient global ischemic rats. A substantial body of experimental data has demonstrated that an increase in ROS levels and subsequent oxidative damage is the leading cause of pathogenesis of transient cerebral ischemia. The extra free radicals directly interact with macromolecules (e.g., proteins, lipids, and DNA) or indirectly by affecting cell signaling pathways and gene regulation [44]. Glutathione, as an intracellular antioxidant, is considered to be an essential cellular protection against oxidative damage [57, 58]. Reduction in GSH levels triggers the release of cytochrome c and induction of cell death signaling [59, 60]. Similar studies have reported that selegiline prevents the reduction of glutathione levels *via* inherent antioxidant properties and increases catalase and superoxide dismutase activities [60, 61]. Our data revealed that the decline in glutathione levels in transient global ischemia is inhibited by selegiline-NBP nanoformulation (0.25-1 mg/kg) in the brain tissue. Nevertheless, selegiline-NBP nanoformulation (0.25 mg/kg) could not normalize the glutathione levels similar to normal rats. It is supposed that decreased levels of glutathione attenuate the immune response against oxidative stress and amplify MDA production in brain tissue. The brain is very rich in PUFA, which is vulnerable to free radical peroxidation. That is the main reason that makes brain especially prone to free radical damage. [62]. Cerebral ischemic animal models have demonstrated deleterious outcomes due to overproduction of MDA, which is the most well-known product of lipid peroxidation, produced from the reactions between free radicals and lipids containing double bound [63]. Similar to our previous study, one investigation suggests the remarkable effectiveness of selegiline in preventing lipid peroxidation after transient global ischemia induction [64]. Interestingly, all of the applied concentrations of selegiline in nanoformulated structures could decrease the amount of MDA to that of normal animals. However, rats treated with nanoformulated selegiline (0.25 mg/kg) could not completely reverse the MDA level to that of the control group.

Another critical parameter and an early event of oxidative stress is protein carbonylation, which is triggered by the reaction of free radicals with proteins as the primary targets of cellular oxidants [29, 65]. Our previous investigation showed an increased level of carbonyl formation in transient global ischemia conditions as a criterion to evaluate the intensity of brain injury [29]. Furthermore, the protein carbonylation level in rats treated with selegiline-NBP nanoformulation (0.5-1 mg/kg) could reach the level of normal rats. Nevertheless, nanoformulated selegiline (0.25 mg/kg) could not completely reverse the amount of protein carbonylation similar to control group levels. These data manifest the antioxidant effects of selegiline to prevent protein oxidation in the brain.

Furthermore, the total antioxidant power of selegiline was determined by FRAP assay, which has been applied to assess the oxidative damage condition [66]. Similar to previous studies in transient global ischemic rats, FRAP levels have been significantly diminished compared to control rats [10]. Besides, the current study confirmed that selegiline nanoformulation (0.5 and 1 mg/kg) effectively returns FRAP levels to that of control rats. However, selegiline nanoformulation (0.25 mg/kg) could not reach the FRAP level to the control level.

## 6. Conclusion

The present study suggested an alternative therapy for developing therapeutic agents in stroke in animal models. We have established selegiline-NBP nanoformulation as a reliable candidate for alternative therapy in transient global ischemia, featuring good biocompatibility, stability, and release profile in an animal model. The finding of this *in vivo* ischemia study suggested that selegiline nanoformulation (0.5-1 mg/kg) could reverse stress oxidative factors including GSH, MDA, protein carbonylation, and FRAP level to that of normal rats. In addition, our data practically confirmed the effectiveness of selegiline-NBP nanoformulation in declining the oxidative stress response. Therefore, we supposed that selegiline-NBP nanoformulation is an appropriate candidate for the treatment of stroke. Nevertheless, future studies are essential to entirely identify the dark concerns on the kinetics of the proposed drug in animal models.

## Figures and Tables

**Figure 1:** Timeline of stroke procedure, treatment behavioral, and biochemical tests. The rats were divided into 7 groups (*n* = 12 animals in each group) and were treated as described in “Materials and Methods.” Each experimental animal group consists of 7-8 animals in behavioral assessments, 3 animals in molecular evaluations, and 2-3 animals in histopathological assays. At the end of treatments, the animals were subjected to the behavioral assessment. In the next step, the effects of drug treatments on the biochemical factors were investigated in the different sets of animals.

**Figure 2:** Scanning electron microscopy (SEM) image of niosomes.

**Figure 3:** The FT-IR spectra of (a) niosomes, (b) niosome-selegiline, and (c) selegiline.

**Figure 4:** Size distribution by intensity of (a) niosomes and (b) niosome-selegiline and zeta-potential of (c) niosomes and (d) niosome-selegiline.

**Figure 5:** (a) Stability curves of niosomes and niosome-selegiline. (b) Rheological behavior of niosomes and niosome-selegiline at room temperature and atmospheric pressure.

**Figure 6:** (a) Percentage of hemolysis induced by niosomes at various concentrations. Cumulative drug release in (b) SIF media (pH 6.80), (c) SGF media (pH 1.2), and (d) buffer solution (pH 7.4).

**Figure 7:** Effects of selegiline on behavioral despair in the NOR test. Values are expressed as the mean ± SD and were analyzed using one-way ANOVA followed by Tukey's post hoc test (*n* = 7 − 8). ^∗^*P* < 0.05, ^∗∗^*P* < 0.01, and ^∗∗∗^*P* < 0.001 compared with control group. ^#^*P* < 0.05 and ^##^*P* < 0.01 and ^###^*P* < 0.001 compared with transient global ischemia rats. “NF = nanoformulated containing NBP; NF+sel = nanoformulated containing NBP+selegiline.”

**Figure 8:** Effects of selegiline on glutathione level in the brain. Values are expressed as the mean ± SD and were analyzed using one-way ANOVA followed by Tukey's post hoc test (*n* = 3). ^∗^*P* < 0.05, ^∗∗^*P* < 0.01, and ^∗∗∗^*P* < 0.001 compared with control group. ^#^*P* < 0.05 and ^##^*P* < 0.01 and ^###^*P* < 0.001 compared with transient global ischemia rats. “NF = nanoformulated containing NBP; NF+sel = nanoformulated containing NBP+selegiline.”

**Figure 9:** Effects of selegiline-NBP nanoformulation on MDA level in the brain. Values are expressed as the mean ± SD and were analyzed using one-way ANOVA followed by Tukey's post hoc test (*n* = 3).^∗^*P* < 0.05, ^∗∗^*P* < 0.01, and ^∗∗∗^*P* < 0.001 compared with control group. ^#^*P* < 0.05 and ^##^*P* < 0.01 and ^###^*P* < 0.001 compared with transient global ischemia rats. “NF = nanoformulated containing NBP; NF+sel = nanoformulated containing NBP+selegiline.”

**Figure 10:** Effects of selegiline on protein carbonylation level in the brain. Values are expressed as the mean ± SD and were analyzed using one-way ANOVA followed by Tukey's post hoc test (*n* = 3). ^∗^*P* < 0.05, ^∗∗^*P* < 0.01, and ^∗∗∗^*P* < 0.001 compared with control group. ^#^*P* < 0.05 and ^##^*P* < 0.01 and ^###^*P* < 0.001 compared with transient global ischemia rats. “NF = nanoformulated containing NBP; NF+sel = nanoformulated containing NBP+selegiline.”

**Figure 11:** Effects of selegiline on FRAP level in the brain. Values are expressed as the mean ± SD and were analyzed using one-way ANOVA followed by Tukey's post hoc test (*n* = 3).^∗^*P* < 0.05, ^∗∗^*P* < 0.01, and ^∗∗∗^*P* < 0.001 compared with control group. ^#^*P* < 0.05 and ^##^*P* < 0.01 and ^###^*P* < 0.001 compared with transient global ischemia rats. “NF = nanoformulated containing NBP; NF+sel = nanoformulated containing NBP+selegiline.”

**Figure 12:** H&E staining images in experimental groups. The effects of different doses of selegiline on neural cell death of hippocampus. Cell death was evaluated *via* hematoxylin-eosin (H&E) staining at 400x magnification. (a):control group; (b) stroke or untreated transient global ischemia rats; (c) nonischemic rats received only noisome+NBP; (d) nonischemic rats received 1 mg/kg of selegiline in niosomal selegiline-NBP structure; (e) stroke rats received selegiline (0.25 mg/kg) in niosomal selegiline-NBP structure; (f) stroke rats received selegiline (0.5 mg/kg) in niosomal selegiline-NBP structure; (g) stroke rats received selegiline (1 mg/kg) in niosomal selegiline-NBP structure. Arrows indicate dead cells.

**Table 1:** Applied statistical models to release data of selegiline.

Function	Equation
*^a^* Zero order	*C* = *C*0 + *K*0*t*
*^b^* First order	ln*C* = ln*C*_0_ + *K*_1_*t*
*^c^* Higuchi	*C* = *K*_*H*_*t*^0.5^
*^e^* Hixson-Crowell	*C*_0_^1/3^ − *C*^1/3^ = *K*_HC_*t*
*^j^* Weibull	*C* = 1 − *e*^−(*t* − *T*_*i*_)^*β*^/*α*^
*^m^* Gompertz	*C* = *e*^−**α**.**e**^−**β**.log(**t**)^^

*^a^ C*_0_ and *C* are the remained amounts of the decoy ODN in the nanocarrier system in the time zero and *t*, respectively; *k*_0_ is the zero-order release constant. *^b^k*_1_ is the first-order release constant.

*^c^ k*_*H*_ is the Higuchi release constant.

*^e^ k*_HC_ is the release constant in Hixson–Crowell model.

*^j^ α* is the scale parameter which defines the time scale of the process; *β* is the shape parameter which characterizes the curve as either exponential (*β* = 1; case 1), sigmoid, S-shaped, with upward curvature followed by a turning point (*β* > 1; case 2), or parabolic, with a higher initial slope and after that consistent with the exponential (*β* < 1; case 3); *T*_*i*_ is the location parameter which represents the lag time before the onset of the dissolution or release process and in most cases will be near zero.

*^m^ α* is the scale factor in the Gompertz model; *β* is the shape factor in the Gompertz model.

**Table 2:** Physicochemical characterization of niosomes and selegiline-niosomes.

Formulation	Conductivity(ms/cm)	pH	RI	% transmittance
Niosomes	1.98	5.41	1.11	42
Selegiline-niosomes	1.32	6.23	1.22	37

**Table 3:** DLS measurement of samples incubated in SGF and SIF media.

Sample	Media	Z-average (nm)		PDI		Zeta-potential (mV)	
		Initial	Final	Initial	Final	Initial	Final
Niosome-selegiline	SGF, pH = 1.2	142.9	279.8	0.346	0.381	-13.8	-8.18
	SIF, pH = 6.8	142.9	290.3	0.346	0.406	-13.8	-7.42

Free niosomes	SGF, pH = 1.2	118.8	231.3	0.254	0.294	-10.5	-5.75
	SIF, pH = 6.8	118.8	286.4	0.254	0.409	-10.5	-4.78

**Table 4:** R2, Akaike's information criterion (AIC) and mean squared error (MSE) parameters from fitting release data of niosome-selegiline and free-selegiline on various models.

Formulation	Niosome-selegiline						Selegiline					
Model	*R* ^2^	AIC	MSE				*R* ^2^	AIC	MSE			
				Parameter						Parameter		
Zero order	0.8152	101.41	9.66	*K*_0_ = 0.538			0.7854	154.95	11.42	*K*_0_ = 0.883		
First order	0.9268	88.43	6.07	*K*_1_ = 0.009			0.8696	103.25	10.31	*K*_1_ = 0.163		
Higuchi	0.9896	61.13	2.29	*K*_*H*_ = 5.47			0.7924	134.01	10.87	*K*_*H*_ = 10.30		
Hixson-Crowell	0.8981	93.07	2.02	*K*_HC_ = 0.003			0.7935	135.55	10.99	*K*_HC_ = 0.011		
Weibull	0.9955	53.26	1.63	*α* = 23.03	*β* = 0.638	*T*_*i*_ = 0.807	0.9626	89.78	6.00	*α* = 1.437	*β* = 0.272	*T*_*i*_ = 1.994
Gompertz	0.9838	69.33	2.97	*α* = 5.15	*β* = 1.07		0.9346	95.59	7.6	*α* = 2.29	*β* = 1.98	

## Data Availability

The data used to support the findings of this study are available from the corresponding author upon request.

## Abbreviations

Sel: L-deprenyl or selegiline
BBB: Blood brain barrier
MOA-B: Monoamine oxidase B
METH: Methamphetamine:
PI3K: Phosphorylation of protein kinase 3
NBP: 4-4-nitrobenzyl pyridine
SEM: Scanning electron microscopy
DLS: Dynamic light scattering:
EC: Electrical conductivity
EE: Entrapment efficiency
PDI: Polydispersity index
PBS: Phosphate-buffered saline
MSE: Mean squared error
AIC: Akaike's information criterion
RBCs: Red blood cells
SDS: Sodium dodecyl sulfate
NIH: National Institutes of Health
NF: Non-ischemic rats received only noisome+ NBP
F+sel: Nonischemic rats received 1 mg/kg of selegiline in niosomal selegiline-NBP structure
Stroke+NF+sel: Stroke rats received selegiline in niosomal selegiline-NBP structure
NOR: Novel object recognition
DI: Discrimination index
GSH: Glutathione
DTNB: 5, 5′-dithiobis-(2-nitrobenzoic acid
TMP: Tetramethoxypropane
MDA: Malondialdehyde
TBA: Thiobarbituric acid
TCA: Trichloroacetic acid
DNPH: 2,4-dinitrophenylhydrazine
FRAP: Ferric-reducing antioxidant power
2-pyridyl: 2,4,6-tris
TPTZ: -1,3,5-triazine
H&E: Hematoxylin and eosin
BSA: Bovine serum albumin
RI: Refractive index
LOD: Refractive index
LOQ: Limit of quantification
SGF: Simulated gastric fluid
SIF: Simulated intestinal fluid.
